The article "Dynamic Surgery Scheduling Based on an Improved Genetic Algorithm" was published in 2021. Journal: J Healthc Eng.

# Dynamic Surgery Scheduling Based on an Improved Genetic Algorithm

**DOI:** 10.1155/2021/1559050

**Published:** 2021-11-22

**Authors:** Bingbing Zhang, Qiang Su

**Affiliations:** School of Economics and Management, Tongji University, Shanghai 200092, China

## Abstract

We formulated a new stochastic programming formulation to solve the dynamic scheduling problem in a given set of elective surgeries in the day of operation. The problem is complicated by the fact that the exact surgery durations are not known in advance. Elective surgeries could be performed in parallel in a subset of operating rooms. The appointment times and assignments of surgeries were planned by an experienced nurses in advance. We present a mathematical model to capture the nature of dynamic scheduling problem. We propose an efficient solution based on an improved genetic algorithm (IGA). Our numerical results showed that dynamic scheduling with the IGA improves the resource utilization as measured by surgeon waiting time and operation room idle time.

## 1. Introduction

High-quality medical resources in China are scarce, and the inefficient use of medical resources makes the scarcity crisis even severer. Surgeries require several medical resources, including operating rooms and human resources [1, 2]. Surgeries are often classified into elective surgery and urgent surgery. Elective surgeries are planned in advance. Compared with elective surgeries, urgent surgeries cannot be planned in advance because of their uncertain nature, and they must be scheduled on a much shorter notice because of the higher priority of urgent surgeries. In many hospitals, urgent surgeries are performed separately. The resources are not shared between elective and urgent surgeries. Urgent surgeries are not taken into consideration in generating a schedule for elective surgeries.

Based on an investigation in Shanghai First People's Hospital, we learned that some operating rooms with special equipment are dedicated to specific types of surgeries. A subset of operating rooms with identical equipment is treated as a common shared resource to serve different elective surgeries. In such a setting, these surgeries can be parallel processed. An experienced nurse must decide on the appointment time for each surgery and the assignment of surgeries to operating rooms prior to the day of surgery. The decisions are made based on estimated surgery durations but are not suitable for practical application. In real situation, the operating process is not as expected. In fact, the duration of surgery is often shortened or lengthened. Therefore, reducing the wasted resource cost incurred by idle operating rooms and waiting surgeons is a challenge. Our study is motivated in part by problems faced by the scheduler who is in charge of elective surgery scheduling.

Based on the actual situation, this paper analyzes the main factors of elective surgery scheduling and studies how to deal with it. The scheduler makes the plan based on limited information in advance. The available information was being continually updated until the day ended. A better schedule is possible when the new information acquired by the scheduler is taken into account. We considered dynamic scheduling with the aim of finding the optimal scheduling strategy. The dynamic surgery scheduling problem was formulated as a multistage decision-making optimization process. At each decision point, we must decide on the sequence and assignment of remaining surgeries according to current status information. The article deals with the simultaneous optimization of both decisions dynamically across multiple operating rooms under uncertainty. Higher resource utilization corresponds to lower wasted cost. The reduction in wasted cost through higher resource utilization can be realized by an optimal schedule. The objective of the model was to minimize the weighted sum of operating room idle time and surgeon waiting time. We analyzed the properties of the dynamic scheduling problem. The mean and standard deviation of surgery duration was estimated based on historical data. The state information of the system was being continually updated until the day ended. Specifically, we rescheduled the remaining surgeries at each decision point based on the current-state information.

The formulated dynamic scheduling problem is NP-hard. Thus, we propose an improved genetic algorithm (IGA) to solve the stochastic optimization model. Holland [3] first proposed a genetic algorithm in 1975. The genetic algorithm has some advantages, such as global optimization, parallel searching, intelligence, and robustness. It has a number of distinct components of the chromosome encoding, the fitness function, the genetic operators, selection, and evolution. The standard component can be improved with due adaptation in an IGA. In this paper, a new chromosome-encoding strategy is proposed according to the nature of dynamic scheduling problem. The current status information of the system at a decision point, including the actual release time of the operating room available, the estimated release times of other operating rooms, and the planned starting times of remaining surgeries, is encoded in a specific chromosome. Each chromosome represents a schedule for the remaining surgeries at that time. The initial population of the chromosomes was randomly generated. Then, a sequence of successive generations evolved. In this way, the IGA ensures the convergence to a best-fitness solution.

The contributions made in this paper are summarized as follows. First, we rescheduled the remaining surgeries by taking into account the new information available at each decision. Second, we constructed a mathematical model of the rescheduling process at any of the decision points. This model was proposed for the joint optimization of surgery sequencing and assignment. Third, we present an IGA that is essential to solve the problem. We proposed a new chromosome-encoding strategy. Each chromosome contains all the updated system information in real time. We also provided a novel way of transforming the solution into the chromosome embodied by code. At last, we quantified the benefit of dynamic scheduling and analyzed the performance of the IGA. The experimental results indicated that our proposed method can obtain better efficiency and global optimization than other common methods.

## 2. Related Work

Khaniyev et al. [4] developed a hybrid heuristic algorithm for the surgery scheduling problem. Their objective was to reduce patient waiting times, operating room idle time, and overtime, and the results showed a 1.22% average performance gap. Lin and Chou [5] proposed a hybrid genetic algorithm that can find near-optimal solutions for the operating room scheduling problem. Zhu et al. [6] proposed a heuristic algorithm incorporated with the grey wolf optimizer with variable neighborhood search to solve operating room scheduling problems. Nasiri et al. [7] developed a fuzzy robust stochastic optimization approach to tackle the multiobjective surgery scheduling model. Hooshmand et al. [8] studied a joint optimization problem of scheduling and rescheduling decisions and developed a genetic algorithm to solve the novel mathematical model. Kamran et al. [9] proposed a sample average approximation method and Benders' decomposition technique to solve the formulated model of two-stage stochastic programming and two-stage chance-constrained stochastic programming. Vali-Siar et al. [10] proposed metaheuristic and heuristic approaches to investigate integrated planning and scheduling problems. The robust counterpart of the problem of allocating operating rooms to surgical cases was solved using a cutting-plane approach [11]. The operating room planning and scheduling problems of a coalition of multiple hospitals were solved by a novel logic-based Benders' decomposition approach [12]. Denton et al. [13] proposed the longest mean service duration fist sequence for sequencing customers. Batun et al. [14] developed a new two-stage stochastic mixed-integer program model to minimize the operation cost under uncertainty. Zhang et al. [15] proposed an algorithm by combining a two-stage stochastic programming approximation and some look-ahead strategies to minimize the total expected cost. Erdogan and Denton [16] scheduled customers dynamically under the condition of first-come-first-served. Erdogan et al. [17] formulated a two-stage stochastic mixed-integer program for the dynamic sequencing and scheduling of appointment requests. Klassen and Yoogalingam [18] developed a simulation optimizing approach to optimize the rules of stochastic appointment scheduling problem. Begen et al. [19] developed a sampling-based approach to determine the planned starting time of each appointment. Hovlid et al. [20] developed a redesigned pathway to reduce the cancellation of planned surgeries. Earlier works on operating room resource utilization concerns service duration under uncertainty [21–23]. Scheduling surgeries is challenging because of the random surgery duration [24–27].

Wasted cost is incurred when operating rooms are idling and surgeons are waiting. Surgeons and other paramedics experience strain differently across the phases of an operation and need effective interventions [28]. Efficient operating room scheduling can lead to cost reduction and utilization improvement [29]. The high utilization of medical resources is necessary to maximize the satisfaction level of patients. Ballestín et al. [30] considered rescheduling patients a few days before the actual period. Some surgeries may be canceled, or other surgeries may be added in the final schedule. The revision of the initial schedule is called rescheduling process. Essen et al. [31] focused on surgery rescheduling by taking into account the preferences and priorities of the stakeholders.

In this article, we focused on surgery scheduling optimization to maximize resource utilization. The study discusses the dynamic scheduling problem of a given set of elective surgeries on the day of execution. We do not consider cancellations of elective surgeries in this article. Our surveys showed that the given set of elective surgeries was scheduled by the scheduler the day before the operation. We focused on a dynamic scheduling strategy to capture the stochastic behavior of surgery durations. The original plan needed to be adjusted accordingly. Thus, we considered rescheduling the updated set of remaining surgeries at each decision point on the course of the day of surgery. We made optimal decisions that involve assignment and sequencing decisions within the operating rooms.

Some previous studies on dynamic scheduling have assumed several fixed rules, including “First Come, First Served (FCFS)”. These studies show that dynamic scheduling decisions make schedules adaptable to variations in a practical situation. In our surveys, we learned that the scheduler reschedules elective surgeries based on a fixed rule during the day of the operation. The survey results provide the best evidence for the practicality and reality of dynamic scheduling. In this paper, we dynamically revised the original schedule through system status updates during the course of the day. Making rescheduling decisions for the remaining surgeries at each decision point is necessary. We described the process of dynamic surgery scheduling as a series of discrete events. Each event represents the rescheduling of the remaining surgeries at each decision point.

## 3. Model Formulation

### 3.1. Problem Description

A given set of elective surgeries are planned prior to the day of surgery. We assume that each surgeon has one surgery a day. The plan includes the start time for each surgery, the assignment of surgeries to operating rooms, and the sequence of surgeries within each operating room. The scheduler is in charge of informing the surgeons of the plan in advance. Then, each surgeon can make his own work schedule for the next day. Therefore, each surgeon is usually not available before the assigned appointment time. These surgeons are assumed to arrive on time to avoid any impact on the availability for their other duties. This original plan is often disrupted throughout the day because of the variability of surgery duration. In this paper, we studied how to simultaneously optimize decisions, including the assignment of surgeries to operating rooms and the sequence of surgeries within each operating room. Our goal was to minimize surgeon waiting time and operating room idle time.

In this section, we formulated the dynamic scheduling problem as a multistage stochastic optimization process.  Figure 1 describes the process of dynamic surgery scheduling in the day of the operation. The discrete nodes on the time axis represent an ordered group of decision points. The *n* − *m* decision points correspond to *n* − *m* discrete events. Each event refers to the rescheduling of the remaining surgeries at each decision point. Remove the last surgery in each operating room from the given set of surgeries. *n* − *m* denotes the number of remaining surgeries. *n* denotes the number of surgeries in the given day, and *m* denotes the number of a subset of interchangeable operating rooms. *t* *=* 0 denotes the starting time of the day, and *t*=*T*_*g*_ denotes the end time of the corresponding surgery *k*(*g*). The latest set of remaining surgeries is rescheduled at each decision point. As a result, a revised schedule of the updated set of remaining surgeries *UA*(*g*) is obtained. The optimization scheme consists of an ordered list of surgeries.

### 3.2. Mathematical Model

#### 3.2.1. Notation

Clinically different types of surgery have different characteristics. Based on the combination of analytical data result and medical information, the distribution of surgery duration is close to a log-normal distribution. *x* denotes any value of time parameter in the equation.

(1) $$\begin{array}{c} P\left(D_{a\left(i\right)}\leq x\right)=F\left(x\right). \end{array}$$

We used the conditional probability model to predict the remaining time for ongoing cases at decision point *g*.

(2) $$\begin{array}{c} P\left(D_{a\left(o\right)}\leq x|D_{a\left(o\right)}>T_{g}-RB_{a\left(o\right)}\right)=\frac{P\left(T_{g}-RB_{a\left(o\right)}<D_{a\left(o\right)}\leq x\right)}{P\left(D_{a\left(o\right)}>T_{g}-RB_{a\left(o\right)}\right)},\;\forall a\left(o\right)\in OG\left(g\right). \end{array}$$

The model is characterized by the following notations in Table 1.

#### 3.2.2. Dynamic Scheduling Model

The dynamic scheduling process is a group of discrete events. Each event represents the procedure of rescheduling the remaining surgeries at the corresponding decision point. The event was formulated as a mathematical model. The optimization goal of the model was to minimize the total wasted cost related to remaining surgeries. The objective function Θ_*g*_ includes the total decision cost related to remaining surgeries at decision point *g*. We aimed to optimize the previous schedule of the remaining surgeries.

(3) $$\begin{array}{c} \Theta_{g}=\min\sum_{a\left(u\right)\in UA\left(g\right)}^{n_{g}}\theta_{a\left(u\right)}. \end{array}$$

Constraint (4) is the cost of scheduling surgery *a*(*u*). The cost *θ*_*a*(*u*)_ includes surgeon waiting time cost and operating room idle time cost. Surgery *a*(*u*) belongs to the set of current remaining surgeries *UA*(*u*). It can be treated as a special stage under the condition, *u* = *g.* The surgery *a*(*g*) is scheduled next to surgery *k*(*g*) , where (*x*)^+^ = max (0, *x*) and *u* is a positive integer.

(4) $$\begin{array}{c} \theta_{a\left(u\right)}=cv{\left(B_{a\left(u\right)}-T_{g}\right)}^{+}+cw{\left(T_{g}-B_{a\left(u\right)}\right)}^{+},\;u=g,\;\forall a\left(u\right)\in UA\left(u\right). \end{array}$$

Constraint (5) defines the cost related to surgery *a*(*u*). Surgery *a*(*u*) is scheduled next to surgery *k*(*u*).

(5) $$\begin{array}{c} \theta_{a\left(u\right)}=cv{\left(B_{a\left(u\right)}-RC_{k\left(u\right)}\right)}^{+}+cw{\left(RC_{k\left(u\right)}-B_{a\left(u\right)}\right)}^{+},\;\forall u>g,\;\forall a\left(u\right)\in UA\left(u\right). \end{array}$$

Constraint (6) defines the updated set of remaining surgeries in real time.

(6) $$\begin{array}{c} UA\left(u\right)=UA\left(u+1\right)\cup a\left(u\right). \end{array}$$

Constraint (7) illustrates the starting time of surgery *a*(*u*).

(7) $$\begin{array}{c} RB_{a\left(u\right)}=\max\left(RC_{k\left(u\right)},B_{a\left(u\right)}\right),\;\forall a\left(u\right)\in UA\left(u\right). \end{array}$$

Constraint (8) illustrates the completion time of surgery *a* (*u*).

(8) $$\begin{array}{c} RC_{a\left(u\right)}=RB_{a\left(u\right)}+D_{a\left(u\right)},\;\forall a\left(u\right)\in UA\left(u\right). \end{array}$$

## 4. Solution Methodology

### 4.1. Problem Structure

In complexity theory, the dynamic scheduling problem is a NP-hard problem. Finding an optimal schedule for such an environment is very difficult because of the extremely large solution space. This problem cannot be solved by general methods in the endurable time. Therefore, heuristic approaches must be used to obtain an optimal approximation solution. An optimal and satisfactory solution for the dynamic scheduling problem is difficult to obtain. We proposed an IGA to solve the problem. The system states at time *T*_*g*_ are characterized by the updated state information. First, the real-time data of the system must be encoded in the genes of an individual. The fitness value of the chromosome is determined by the linear order of genes along a chromosome. The ones with least fitness have a greater chance of selection. We provided the chromosome-coding schemes and fitness function to design and realize the surgery rescheduling system. Matrix **L**_*g*_ containing (*n* − *g*+1)^2^ elements is generated at decision point *g*. Each element represents the length of a gene fragment. *g* denotes the number of completed surgeries. In this square matrix, the number of rows is equal to the number of genes. The number of genes is (*n* − *g*+1); the number of remaining surgeries is (*n* − *m* − *g*+1); and the number of identical operating rooms is *m.* The proposed formulas are listed below for evaluating the length of different gene fragments.

(9) $$\begin{array}{c} l_{ri}\left(g\right)={\left(B_{i}-T_{g}\right)}^{+},\;r=r\left(g\right),\\ l_{ri}\left(g\right)={\left(B_{i}-t_{r}\left(g\right)\right)}^{+},\;\forall r\in R,\;r\neq r\left(g\right),\\ l_{ij}={\left(B_{j}-\left(B_{i}+D_{i}\right)\right)}^{+},\;\forall i\in I,\\ L_{g}=\left[\begin{array}{cccccc} l_{11} & \cdots & l_{1m} & l_{1\left(m+1\right)} & \cdots & l_{1\left(n-g+1\right)}\\ \cdots & \cdots & \cdots & \cdots & \cdots & \cdots \\ l_{m1} & \cdots & l_{mm} & l_{m\left(m+1\right)} & \cdots & l_{m\left(n-g+1\right)}\\ l_{\left(m+1\right)1} & \cdots & l_{\left(m+1\right)m} & l_{\left(m+1\right)\left(m+1\right)} & \cdots & l_{\left(m+1\right)\left(n-g+1\right)}\\ \cdots & \cdots & \cdots & \cdots & \cdots & \cdots \\ l_{\left(n-g+1\right)1} & \cdots & l_{\left(n-g+1\right)m} & l_{\left(n-g+1\right)\left(m+1\right)} & \cdots & l_{\left(n-g+1\right)\left(n-g+1\right)} \end{array}\right]. \end{array}$$

### 4.2. Improved Genetic Algorithm

The IGA with a special chromosome-coding scheme was applied to the dynamic scheduling problem in multiple operating room setting. The crucial part of the proposed method is how to transform the solution into the chromosome embodied by code.  Figure 2 depicts an example with three operating rooms and eight surgeries for the first decision point. A randomly generated chromosome represents a schedule of the joint optimization of the assignment and the sequencing of the remaining surgeries at the decision point.

We proposed an IGA for rescheduling the remaining surgeries at time *T*_*g*_. The main steps of the proposed method are as follows:

IGA

  Step 1 (initialization): Set the population number (*Q*), gene number (*n* − *g*+1), iteration number (DC), selection probability (*P*_s_), crossover probability (*P*_c_), and mutation probability (*P*_m_)
  Step 2. Randomly generate the initial population of chromosomes; provide the chromosome coding schemes *l*_*ri*_(*g*)=(*B*_*i*_ − *T*_*g*_)^+^,  *r*=*r*(*g*)*l*_*ri*_(*g*)=(*B*_*i*_ − *t*_*r*_(*g*))^+^,  ∀ *r* ∈ *R*,  *r* ≠ *r*(*g*)*l*_*ij*_=(*B*_*j*_ − (*B*_*i*_+*D*_*i*_))^+^,  ∀ *i* ∈ *I*
  Step 3. Set fitness function as an indicator. Calculate the length of each chromosome in the population len(*i*, 1)=length(*L*_*g*_, population(*i*, :)); calculate the fitness of each chromosome fit(*i*, 1)=fitness(len(*i*, 1), *a*, maxlen, minlen)
  Step 4. Conserve the best individual: [len_*m*, len_index]=min(len_1)
  Step 5. Design the genetic operators: *P*_s_, *P*_c_, and *P*_m_
  Step 6. Generate a new generation of individuals as the successor population
  Step 7. Repeat steps 3–6 until the loop termination condition has been reached. The terminating condition is the fixed number of iterations (DC) reached.
  Step 8. End

## 5. Results and Discussion

### 5.1. Results

This section presents the results of the experiments to illustrate the structure of the optimal schedule for a specific example and evaluate the performance of the proposed method in different problem instances. The proposed algorithm was coded in MATLAB R2013a. The experiments were conducted on Intel Core i7 PC at 2.40 GHz with 4 GB memory. The instances of this paper were derived from field observations in Shanghai First People's Hospital. First, we considered a specific instance with a given set of 12 different general surgeries on the day of service. Three operating rooms were interchangeable and allotted for general surgeries.

The following are the results of the performance evaluation of the proposed method on the instance. The behavior of the graphs is shown in Figure 3.  Figure 3(a) shows the experimental results at decision point, *g*=1. The fitness values of individuals reflect the objective function values. The optimal fitness curve includes points, which represents the fitness value of the best chromosome in every generation of the evolution process. The results in Figure 3 indicate that the algorithm guarantees global convergence and improves the converging rate and stability.

The optimal solution of the instance is presented in Table 2. The results are presented in terms of optimal individual, minimum and reference fitness values, and CPU time for the instance. Table 2 shows the optimal schedule of the remaining surgeries at each decision point. The optimal individual that evolved at decision point *g* represents the optimal schedule obtained for three operating rooms. The set of remaining surgeries was updated in real time. Specifically, the order of genes along a chromosome represents the optimal schedule of remaining surgeries. The algorithm has great ascendancy because its ability for the global search of optimal individual is powerful. The experiment results indicated that the algorithm can obtain the optimal schedule in a short time.

### 5.2. Discussion

This section presents the evaluation results of the benefit of solving the dynamic scheduling problem compared with solving the static scheduling problem. The relative benefit provides a measure of the value of dynamic scheduling related to the commonly used approach in scheduling practice.

An experiment was performed to evaluate the changes in relative benefit according to the workload of the system (WS) and the variance of surgery durations (VD).  Table 3 shows the minimum, maximum, and average relative benefits for these runs. According to the results in Table 3, the relative benefit decreases as the WS increases. Experimental results indicated that our proposed method still has a better performance than static planning in high-workload cases. The relative benefit increases as VD increases (Table 3). The results illustrated that our method is appropriate for high-uncertainty cases. Therefore, our proposed method has practicality, reliability, and stability. A series of revised schedules were sequentially made throughout the day by taking into account the changes in system information. Therefore, the optimal schedule obtained is flexible.

In our next experiment, we compared dynamic scheduling based on IGA with some other methods. We evaluated the computational performance of our proposed method.

Table 4 presents the optimality gaps. Our method has superior performance in rescheduling surgeries. The results imply that our proposed method outperforms some other methods. The proposed method has good convergence and excellent robustness. Dynamic scheduling based on a fixed discipline focuses on the decision-making costs of a single stage. Our method takes into account the decision-making costs of all the remaining stages. The optimal schedule depends on many decisions, most of which have an effect on one another.

Furthermore, we compared the proposed IGA with local search algorithms. A local search algorithm is a common approximate search algorithm. Many previous studies applied this heuristic algorithm in optimization problems.

We tested 30 instances and randomly selected the results of 3 instances of three operating rooms problem and 3 instances of six operating rooms. Optimality gap provides a measure of the performance of the IGA relative to local search heuristic algorithm in surgery rescheduling. According to the results presented in Table 5, optimality gap increases as the number of operating rooms increases. Our method has better performance than the local search algorithm. Compared with the local search heuristic algorithm, the proposed method can be applied to optimize global parameters. The results showed that our method has a potential to find a better solution. The method can work at a blindingly fast speed by adopting an adaptive parallel search strategy.

## 6. Conclusions

In this paper, we describe the dynamic scheduling process as a series of discrete events. Each event represents the procedure of rescheduling the remaining surgeries at each decision point. We formulated the rescheduling process as a multistage stochastic optimization model. The dynamic scheduling problem has an extremely large state space; thus, we proposed the IGA to solve the problem. The chromosome-coding schemes and fitness function were provided to design and realize the surgery rescheduling system. Numerical results show that our proposed method has superior performance compared with some common scheduling approaches. The results of different instances also show that our proposed method has good convergence and excellent robustness. The solution space increased with the enlargement of the scale of the problem. We found that the proposed method can converge into a globally optimal solution compared with traditional algorithms in large-scale problems.

We also observed that the estimation of surgery durations influences the schedule optimization, especially in high-workload instances. Moreover, estimating the service times of the remaining surgeries is a challenge. Our method has its limitation. Future studies should consider historical sample sizes with estimated means and variances in log scale. There are some limitations of our research, which present opportunities for future work. For example, our proposed method should be robust to a disruption from a single urgent surgical case. There may be scenarios need to be considered such as no urgent surgeries, single urgent surgery, and multiple urgent surgeries. In the future work, we will focus on the study of global scheduling strategy to improve the quality of medical services and patient satisfaction.

## Figures and Tables

**Figure 1:** Dynamic surgery rescheduling process.

**Figure 2:** Translation process of chromosome encoding.

**Figure 3:** Results of the instances: (a) *g*=1, (b) *g*=2, (c) *g*=3, (d) *g*=4, (e) *g*=5, (f) *g*=6.

**Table 1:** Parameters and description.

Parameter	Description
*UA*(*u*)	Set of remaining surgeries
*a*(*u*)	*u*th surgery to be performed next
*k*(*u*)	*u*th completion surgery
*D*_*a*(*u*)_	Estimated duration of surgery
*B*_*a*(*u*)_	Arrival time of surgeon
*RB*_*a*(*u*)_	Starting time of surgery
*RC*_*a*(*u*)_	Completion time of surgery
*θ*_*a*(*u*)_	Decision-making cost of surgery
*n*	Number of surgeries
*m*	Number of operating rooms
*g*	Index of decision points
*n*_*g*_	Number of remaining surgeries at the decision point
*cv*	Unit idle time cost of operating room
*cw*	Unit waiting time cost of surgeon
*R*	Set of operating rooms
*r*	Index of operating rooms

**Table 2:** Optimal solution of the instance.

	Optimal individual	Fitness value		CPU time (sec)
		Min	Ref	
*g*=1	**1**-4-7-10-**2**-5-9-12-**3**-6-8-11	110	257.61	101.50
*g*=2	**1**-6-7-11-**2**-9-12-**3**-4-8-10	196	505.40	101.28
*g*=3	**1**-7-12-**2**-9-11-**3**-4-8-10	204	611.42	101.32
*g*=4	**1**-8-12-**2**-7-10-**3**-9-11	56	678.95	101.16
*g*=5	**1**-8-12-**2**-10-**3**-9-11	258	661.81	101.18
*g*=6	**1**-11-**2**-10-**3**-9-12	132	462.78	101.24

**Table 3:** Results for the problem instances.

Workload	Variance	Relative benefit (%)		
		Min.	Max.	Average
WS < 100%	VD < 25%	24.25	41.74	29.06
	VD > 25%	27.56	49.00	33.45

WS > 100%	VD < 25%	12.53	26.81	16.62
	VD > 25%	16.85	35.17	23.90

**Table 4:** Comparison of our method with other methods.

Method	Optimality gap (%)
The longest mean service duration first sequence [13]	9.5
Two-stage stochastic programming approximation [15]	2.7
First-come-first-served strategy [16]	6.0

**Table 5:** Comparison of the IGA with local search algorithm for instances.

	3 operating rooms			6 operating rooms		
Instance no.	1	2	3	4	5	6
Optimality gap (%)	6.4	5.1	9.0	12.3	15.6	9.8

## Data Availability

The data utilized to support the findings are available from the corresponding author on reasonable request.
